This article has been retracted.

# GEO Database Screening Combined with In Vitro Experiments to Study the Mechanism of hsa_circ_0003570 in Infantile Hemangiomas

**DOI:** 10.1155/2022/5643742

**Published:** 2022-04-28

**Authors:** Yu Tian, Shihao Zhuang, Jiantao Zhang, Tonghui You, Zihang Xu, Wanli Yang, Bin Hao, Weifeng Wang, Tao Yang

**Affiliations:** ^1^Shanxi Bethune Hospital, Shanxi Academy of Medical Sciences, Tongji Shanxi Hospital, Third Hospital of Shanxi Medical University, Taiyuan 030032, China; ^2^Fujian Children's Hospital; Fujian Maternity and Child Health Hospital, Affiliated Hospital of Fujian Medical University, Fuzhou 350000, China; ^3^Third Hospital of Shanxi Medical University, Shanxi Bethune Hospital, Shanxi Academy of Medical Sciences, Tongji Shanxi Hospital, Taiyuan 030032, China; ^4^Department of Central Laboratory, Shanghai Tenth People's Hospital, Tongji University School of Medicine, Shanghai 200435, China; ^5^Department of Clinical Laboratory Medicine, Longhua Hospital Shanghai University of Traditional Chinese Medicine, Shanghai 200030, China

## Abstract

**Objective:**

In this study, we screened out a type of differentially expressed circular RNA in infantile hemangioma (IH) cells and analyzed the mechanism in the malignant biological behavior of IH.

**Methods:**

Based on the GSE98795, GSE100682, and GSE43742 datasets, differential expression analysis of circRNAs, microRNAs, and mRNAs was performed. The relative expression level of RNA was detected by quantitative real-time polymerase chain reaction (qRT-PCR). MTT assay, Transwell, flow cytometry analysis, and western blot were used to study the effects of hsa_circ_0003570, hsa-miR-138-5p, and RGS5 on the proliferation and apoptosis of hemangioma endothelial cells (HEMECs).

**Results:**

The hsa_circ_0003570 and *RGS5* mRNA were upregulated in HEMECs, but hsa-miR-138-5p was downregulated. Silencing of hsa_circ_0003570 inhibited the proliferation of HEMECs and promoted the apoptosis of HEMECs. The malignant biological behaviors of hsa_circ_0003570 on the proliferation and apoptosis of HEMECs were reversed by hsa-miR-138-5p. Hsa_circ_0003570 acted as the ceRNA of hsa-miR-138-5p and upregulated the expression of RGS5. Silencing of RGS5 inhibited the proliferation, migration, and invasion of HEMECs and promoted apoptosis.

**Conclusion:**

Hsa_circ_0003570 promotes IH cell proliferation and inhibits IH cell apoptosis through hsa-miR-138-5p/RGS5 axis.

## 1. Introduction

IH is a kind of soft tissue benign tumor in infants and young children [1]. The incidence was about 3 to 5% and increased in recent years [2–4]. Although most IH are benign and have a self-limiting course, about 10% of IH can grow rapidly and cause serious complications, such as bleeding, ulceration, and impaired appearance, requiring early active intervention [5, 6].

Current research evidence showed that the occurrence and development of IH were jointly regulated by exogenous factors such as tissue hypoxia, developmental defects, and endogenous genes [6–10]. Noncoding RNA (ncRNA) occupies 98%-99% of the human genome transcript, and it has been confirmed that it can affect the occurrence and development of various diseases by regulating gene expression [11, 12].

Circular RNA is a special type of ncRNAs, which is formed by alternative splicing of precursor mRNA. It is a closed-ring structure with the 3′ and the 5′ ends connected by a covalent bond [13]. circRNA has the characteristics of high abundance, high stability, sequence conservation, tissue and developmental stage specificity, etc., and it is an important regulatory factor in the occurrence and development of diseases [14, 15]. The current findings suggested that circRNAs could act as a molecular sponges for microRNAs, competitive endogenous RNAs (ceRNAs), and binding microRNAs and preventing them from binding to downstream target genes, thereby regulating gene expression [16]. In addition, circRNA can also play a role in transcription and splicing regulation [17], circRNA-protein interaction [18, 19], and translation protein [20].

Both angiogenesis and revascularization are involved in the occurrence of IH, but the specific mechanism needs to be further studied [21]. A feasible approach is to screen differentially expressed genes, microRNAs, and circRNAs in IH and study how they function in the occurrence of IH, which may provide new evidence for understanding the mechanism of IH.

In this study, we selected hsa_circ_0003570, hsa-miR-138-5p, and RGS5 for research by analyzing the differential transcription profiles of GSE98795, GSE100682, and GSE43742 datasets. Through bioinformatics tools, it was found that hsa_circ_0003570 and hsa-miR-138-5p as well as hsa-miR-138-5p and RGS5 had complementary pairing sequences. Therefore, we speculate that the hsa_circ_0003570/hsa-miR-138-5p/RGS5 axis may play a key role in the occurrence of IH. To prove our hypothesis, we studied the role of hsa_circ_0003570, hsa-miR-138-5p, and RGS5 in the malignant biological behavior of IH in the hemangioma endothelial cells (HEMEC) model, and through our research results, we provided a new direction for the treatment of IH. The flow chart was shown in Figure 1.

## 2. Materials and Methods

### 2.1. Datasets

The GSE98795 dataset [22] was used for differential expression analysis of circRNAs, the GSE100682 dataset was for microRNAs, and the GSE43742 dataset was for mRNAs, all these datasets were obtained from GEO DataSets (https://www.ncbi.nlm.nih.gov/gds/).

### 2.2. Cell Culture

Human dermal microvascular endothelial cells (HDMVECs) and HEMECs were cultured in DMEM (Invitrogen, Carlsbad, CA, USA) with 10% FBS (Gibco, Carlsbad, CA, USA) and incubated in a humidified atmosphere containing 5% CO_2_ at 37°C.

### 2.3. Cell Transfection

The hsa_circ_0003570 small interfering RNA (named si-hsa_circ_0003570)-1, 2, 3 and si-no temple control (NC), hsa-miR-138-5p mimic, hsa-miR-138-5p inhibitor, hsa-miR-NC, pGL3-hsa_circ_0003570 wild-type (WT), pGL3-hsa_circ_0003570 mutant (MUT), pGL3-RGS5 wild-type (WT), pGL3-RGS5 mutant (MUT), short hairpin RNA no temple control (sh-NC), and sh-RGS5 were synthetized by GenePharma (Shanghai, China). The recombinant plasmid was transfected into HEMECs with Lipofectamine 2000 (Invitrogen, Carlsbad, CA). QRT-PCR and western blot were used to detect transfection efficiency. In order to screen the stable transfected HEMECs with the highest silencing efficiency, HEMECs were divided into 5 groups: control, si-NC, si-hsa_circ_0003570-1, and si-hsa_circ_0003570-2, si-hsa_circ_0003570-3. In order to analyze the role of hsa-miR-138-5p in hsa_circ_0003570-silenced HEMECs, HEMECs were divided into 5 groups: control, si-NC, si-hsa_circ_0003570, si-hsa_circ_0003570+hsa-miR-138-5p inhibitor, and hsa-miR-138-5p inhibitor. In dual luciferase assay, HEMECs were divided into 8 group: hsa-miR-NC+pGL3-hsa_circ_0003570 WT, hsa-miR-NC+pGL3-hsa_circ_0003570 MUT, hsa-miR-138-5p mimic+pGL3-hsa_circ_0003570 WT, hsa-miR-138-5p mimic+pGL3-hsa_circ_0003570 MUT, hsa-miR-NC+pGL3-RGS5 WT, hsa-miR-NC+pGL3-RGS5 MUT, hsa-miR-138-5p mimic+ pGL3-RGS5 WT, and hsa-miR-138-5p mimic+pGL3-RGS5 MUT. In order to study the effect of RGS5 silencing on the malignant biological behavior of HEMECs, HEMECs were divided into 3 group: control, sh-NC, and sh-RGS5. All samples were run in triplicate.

### 2.4. Quantitative Real-Time Polymerase Chain Reaction (qRT-PCR)

Total RNA was isolated from HEMECs with Trizol reagent (Life Technologies Corporation, Carlsbad, CA, USA). One-Step SYBR PrimeScript RT-PCR Kit (TakaraBio, Inc., Japan) was used to detect the expression of hsa_circ_0003570, hsa-miR-138-5p, and *RGS5* mRNA. The PCR conditions were 95°C for 5 min, then 95°C for 10s, 58°C for 20s, and 72°C for 30s, and repeated for 45 cycles. The primer sequences of hsa_circ_0003570 were 5′-AACTTGTGTCCAGAAAGTGCTT-3′(forward); 5′-AAGATGGCACAGCACACGC-3′ (reverse). Hsa-miR-138-5p: 5′-GCCGAGCTGGTGTTGTGAAT-3′ (forward); 5′-GTGCAGGGTCCGAGGTATTC-3′ (reverse). *RGS5* mRNA: 5′-AAGATGGCTGAGAAGGCAAA-3′ (forward); 5′-TCAGGGCATGGATTCTTTTC-3′ (reverse). U6: 5′-AACGCTTCACGAATTTGCGT-3′ (forward); 5′-CTCGCTTCGGCAGCACA-3′ (reverse). The relative expression level was calculated by 2^-∆∆Ct^. All samples were run in triplicate.

### 2.5. MTT Assay

After 24 h of transfection, HEMECs were digested with trypsin. HEMECs were seeded 5 × 10^3^ cells/well in 96-well. After incubated for 0, 24, 48, and 72 h, MTT (Sigma-Aldrich, St. Louis, MO, USA) was added to every well and incubated for 4 h. Then, 150 *μ*l of DMSO was added into each well and mixed for 10 min. The absorbance at 490 nm was detected at 0 h, 24 h, 48 h, and 72 h. All samples were run in triplicate.

### 2.6. Transwell Assay

HEMECs were harvested after 24 h transfection. Migration and invasion of transfection HEMECs were detected by Transwell assay. The specific experimental procedures refer to the research of Zhou et al. [23]. All samples were run in triplicate.

### 2.7. Dual Luciferase Assay

The sequence of hsa_circ_0003570 and RGS5 and their mutant sequence of hsa-miR-138-5p binding sites were synthesized by PCR and cloned into pGL3-Basic (Promega, Madison, WI, USA). The pGL3-hsa_circ_0003570 WT or pGL3-hsa_circ_0003570 MUT and hsa-miR-138-5p mimic (or has-miR-NC) were cotransfected into HEMECs, and pGL3-RGS5 WT, pGL3-RGS5 MUT, and hsa-miR-138-5p mimic (or has-miR-NC) were cotransfected into HEMECs. The luciferase activities were detected by the Dual-Lucifer Reporter Assay System 48 h later, and the relative luciferase activity was calculated by normalizing to Renilla luciferase activity. All samples were run in triplicate.

### 2.8. Western Blot

Total protein in HEMECs was separated by SDS-PAGE. The proteins were transferred onto polyvinylidene fluoride (PVDF) membranes from SDS-PAGE. Then incubated the PVDF membrane with rabbit anti-RGS5 (ab96799, 1: 1500, Abcam, Cambridge, MA) primary antibodies at 4°C for 12 h-16 h, then incubated at room temperature for 2 hours with secondary antibody. RGS5 protein was visualized using ECL Plus Western blotting Detection Reagents (Millipore, Billerica, MA).

### 2.9. Statistical Analysis

Discontinuous variables should be presented as percentages, while continuous variables in normal distribution should be described as mean ± standard deviation (SD) or else reported as median (range). Variance homogeneous and normal distributed continuous variables could be compared by student *t*-test, otherwise, the Mann–Whitney *U*-test or Kruskal-Wallis *H*-test would be used, *p* < 0.05 indicated that the difference was statistically significant. The statistical analyses were presented by GraphPad Prism 8.0 (GraphPad Software, San Diego, CA).

## 3. Results

### 3.1. Human Infantile Hemangioma Endothelial Cells (HEMECs) from Proliferating Tumor Transcriptome Analysis

Based on the GEO database, the GSE98795 dataset was selected for differential expression analysis of circRNAs in this study. A total of 234 circRNAs were upregulated, and 374 circRNAs were downregulated (Supplementary Table 1, FC (abs) cut-off value 1.0). The GSE100682 dataset was selected for differential expression analysis of microRNAs. The results showed that 329 microRNAs were upregulated and 337 microRNAs were downregulated (Supplementary Table 2, logFC cut-off value 1.0). The GSE43742 dataset was selected for differential expression analysis of mRNAs. The results showed that 23 mRNAs were upregulated and 25 mRNAs were downregulated (Supplementary Table 3, logFC cut-off value 2.0).

In this study, we chose hsa_circ_0003570, hsa-miR-138-5p, and RGS5 for research, because according to the Encyclopedia of RNA Interactomes (ENCORI) [24], analysis results showed that both hsa_circ_0003570 and RGS5 had binding sites to hsa-miR-138-5p (Figure 2(a)). We detected the expression levels of hsa_circ_0003570, hsa-miR-138-5p, and *RGS5* mRNA in human dermal microvascular endothelial cells (HDMVECs) and HEMECs, respectively. The results showed that hsa_circ_0003570 and *RGS5* mRNA were upregulated in HEMECs, and hsa-miR-138-5p was downregulated, the differences were significant (*p* < 0.05, Figure 2(b)).

### 3.2. Silencing of hsa_circ_0003570 Inhibited the Proliferation and Promoted Apoptosis of HEMECs

We found that hsa_circ_0003570 was highly expressed in HEMECs according to the GSE98795 dataset, indicating that hsa_circ_0003570 might have carcinogenic effects. In order to analyze the role of hsa_circ_0003570 in the biological behavior of HEMECs, we constructed three groups of hsa_circ_0003570 small interfering RNAs (siRNAs) to silence hsa_circ_0003570, respectively, named si-hsa_circ_0003570-1, si-hsa_circ_0003570-2, and si-hsa_circ_0003570-3, and the no template control (si-NC) and the nontransfection group (control) were used as controls.

We chose si-hsa_circ_0003570-1 (named si-hsa_circ_0003570) with the highest silencing efficiency for subsequent research (Figure 3(a)). Compared with the control, the cell proliferation ability of si-hsa_circ_0003570 transfected with HEMECs decreased significantly (*p* < 0.05, Figure 3(b)). The migration and invasion capabilities of HEMECs were significantly reduced after transfection with si-hsa_circ_0003570 (*p* < 0.01, Figures 3(c) and 3(d)). The apoptosis rate of HEMECs after transfection with si-hsa_circ_0003570 was significantly higher than that of the control (*p* < 0.001, Figure 3(e)). The results indicated that silencing of hsa_circ_0003570 inhibited the proliferation and promoted apoptosis of HEMECs.

### 3.3. The Effect of hsa_circ_0003570 on the Malignant Biological Behavior of HEMECs Could Be Reversed by hsa-miR-138-5p

To further analyze the role of hsa-miR-138-5p in hsa_circ_0003570-silenced HEMECs, the expression level of hsa_circ_0003570 and hsa-miR-138-5p in HEMECs transfected with control, si-NC, si-hsa_circ_0003570, si-hsa_circ_0003570+hsa-miR-138-5p inhibitor, and hsa-miR-138-5p mimic was shown in Figure 4(a). The results showed that compared with the control, the proliferation ability of HEMECs was significantly decreased after transfection with si-hsa_circ_0003570 and hsa-miR-138-5p mimic (*p* > 0.05), no significant change in the proliferation ability after si-hsa_circ_0003570+hsa-miR-138-5p inhibitor transfection significantly (*p* > 0.05, Figure 4(b)). After transfection with si-hsa_circ_0003570 and hsa-miR-138-5p mimic, the migration and invasion capabilities of HEMECs were significantly reduced (*p* < 0.05), but HEMECs transfected with si-hsa_circ_0003570+hsa-miR-138-5p inhibitor were not (*p* > 0.05, Figures 4(c) and 4(d)).

The apoptotic rate of HEMECs after transfection with si-hsa_circ_0003570 and hsa-miR-138-5p mimic was significantly higher than the control (*p* < 0.05), but there was no significant change in the apoptosis rate of HEMECs after cotransfection with si-hsa_circ_0003570+hsa-miR-138-5p inhibitor (*p* > 0.05, Figure 4(e)). The above results indicated that the effect of hsa_circ_0003570 on the malignant biological behavior of HEMECs could be reversed by hsa-miR-138-5p.

### 3.4. Hsa_circ_0003570 Upregulated the Expression of RGS5 through Sponging hsa-miR-138-5p

According to the prediction results of ENCORI, both hsa_circ_0003570 and *RGS5* had binding sites with hsa-miR-138. The wild-type luciferase vector (pGL3-hsa_circ_0003570 WT, pGL3-RGS5 WT) and mutant luciferase vector (pGL3-hsa_circ_0003570 MUT, pGL3-RGS5 MUT) were constructed, respectively (Figures 5(a) and 5(c)). Next, hsa-miR-138-5p mimic and pGL3-hsa_circ_0003570 WT, pGL3-hsa_circ_0003570 MUT, pGL3-RGS5 WT, and pGL3-RGS5 MUT were transfected into HEMECs, respectively. According to the results, the luciferase activity of hsa-miR-138-5p mimic and pGL3-hsa_circ_0003570 WT, hsa-miR-138-5p mimic, and pGL3-RGS5 WT was significantly reduced after transfection, while hsa-miR-138-5p mimic and pGL3-hsa_circ_0003570 MUT, hsa-miR-138-5p mimic, and pGL3-RGS5 MUT did not change significantly after transfection (Figures 5(b) and 5(d)). Then, the control, NC, si-hsa_circ_0003570, hsa-miR-138-5p mimic, si-hsa_circ_0003570+hsa-miR-138-5p inhibitor, and hsa-miR-138-5p inhibitor were transfected into HEMECs, respectively, and the expression levels of hsa_circ_0003570, hsa-miR-138-5p, and *RGS5* mRNA were detected by qRT-PCR. The results showed that compared with control, the expression level of hsa-miR-138-5p increased after transfection of si-hsa_circ_0003570 or hsa-miR-138-5p mimic, while the expression level of *RGS5* mRNA was inhibited.

After transfection with hsa-miR-138-5p inhibitor, the expression level of hsa-miR-138-5p was significantly reduced, and *RGS5* mRNA was increased. After transfection with si-hsa_circ_0003570+hsa-miR-138-5p inhibitor, the expression level of hsa-miR-138-5p decreased, but the expression level of *RGS5* mRNA did not change significantly (Figure 5(e)). Western blot results showed that compared with control, the expression of RGS5 protein was significantly reduced after transfection with si-hsa_circ_0003570 or hsa-miR-138-5p mimic. After transfection with hsa-miR-138-5p inhibitor, the expression level of RGS5 protein increased. And RGS5 expression level did not change significantly when transfected with si-hsa_circ_0003570+hsa-miR-138-5p inhibitor (Figure 5(f)). These results indicated that hsa_circ_0003570, as the ceRNA of hsa-miR-138-5p, upregulated the expression of RGS5.

### 3.5. RGS5 Knockdown Inhibited the Proliferation and Promoted Apoptosis of HEMECs

In order to further study the effect of RGS5 on the malignant biological behavior of HEMECs, we constructed a short hairpin RNA (shRNA) (sh-RGS5) targeting RGS5 to silence the expression of *RGS5* gene. The results of qRT-PCR and western blot showed that we successfully constructed RGS5-silenced HEMECs (Figures 6(a) and 6(b)). The results of the MTT assay showed that compared with the control, the cell proliferation ability of HEMECs transfected with sh-RGS5 was significantly reduced (*p* < 0.05, Figure 6(c)). Results showed that the migration and invasion capabilities of HEMECs were significantly reduced after sh-RGS5 transfection (*p* < 0.01, Figures 6(d) and 6(e)). The apoptosis rate of HEMECs after sh-RGS5 transfection was significantly higher than the control (*p* < 0.001, Figure 6(f)). These results indicated that RGS5 knockdown inhibited the proliferation and promoted apoptosis of HEMEC.

## 4. Discussion

Circular RNA is a kind of ncRNA molecule with a special closed circular structure. It has the characteristics of high stability, conservation, and tissue specificity. In recent years, it has become a hot spot in the field of ncRNA research [15, 25–27]. Studies have found that circRNAs are differentially expressed in tumors [28, 29], cardiovascular diseases [30–32], nervous system, and other diseases [33, 34] and affect the occurrence and development of diseases through various mechanisms.

There are many differentially expressed circRNAs in hemangioma. For example, Yuan et al. [35] found that circAP2A2 can promote the proliferation and invasion of IH by regulating the miR-382-5p/VEGFA axis. Through RNA-Seq research, Li et al. [36] found that among 9811 identified circRNAs, 249 candidate genes were differentially expressed, including 124 upregulated and 125 downregulated circRNAs. The study of these circRNAs is of great value for the prevention and treatment of IH and explaining the mechanism of IH occurrence and development.

In this study, we combined with the results of the GSE98795 dataset [22] and found that hsa_circ_0003570 in HEMECs was upregulated. In order to further verify the possible mechanism of hsa_circ_0003570 in the occurrence and development of IH, small interfering RNA were used to knock down the expression level of hsa_circ_0003570 in HEMECs. The results showed that silencing of hsa_circ_0003570 inhibited the proliferation and promoted apoptosis of HEMECs. This result indicated that hsa_circ_0003570 might be the oncogene of IH.

A lot of research evidence showed that circRNAs could be used as ceRNA to regulate gene expression and participated in the occurrence of diseases [16, 37, 38]. Therefore, we analyzed the data in the GSE100682 dataset, combined with target prediction information, and selected hsa-miR-138-5p for research. Studies had shown that hsa-miR-138-5p could promote the angiogenesis of HUVECs infected by human cytomegalovirus (HCMV) through activating SIRT1-p-STAT3 approach [39]. This showed that hsa-miR-138-5p played an important role in angiogenesis. In this study, we found that the expression level of hsa-miR-138-5p in HEMECs was significantly downregulated, and hsa-miR-138-5p could reverse the effect of hsa_circ_0003570 on the proliferation, migration, invasion, and apoptosis of HEMECs. Therefore, we speculated that hsa-miR-138-5p might mediate the regulation of hsa_circ_0003570 on the expression of key downstream genes.

We further studied in the GSE43742 dataset and found that the expression of 23 mRNAs was upregulated and 25 mRNAs downregulated. Combined with the results of target prediction, we found that the *RGS5* gene was upregulated HEMECs, which was consistent with the study by Stiles et al. [40]. In addition, the *RGS5* gene also has a binding site for hsa-miR-138-5p. Further studies had shown that silencing *RGS5* inhibited the proliferation and promoted apoptosis of HEMECs. This showed that RGS5 may be the oncogene of IH. The luciferase assay experiment confirmed that hsa_circ_0003570, as the ceRNA of hsa-miR-138-5p, upregulated the expression of RGS5. Therefore, we speculate that hsa_circ_0003570 participates in the regulation of the malignant biological behavior of IH through hsa-miR-138-5p/RGS5 axis and is expected to become a potential target for IH therapy.

Our research has some shortcomings that need to be improved. First of all, there is a lack of research evidence support for tissue samples, our findings have only been validated in HEMEC cell line, and further study in tissue samples and other cell lines are needed to solve these problems. In fact, the results of in vitro need to be confirmed in in vivo. In addition, the mechanism of IH is relatively complicated, and there may be a large number of other pathways involved to study.

## 5. Conclusion

In conclusion, our research confirmed that hsa_circ_0003570 regulated the proliferation, migration, and invasion of IH through hsa-miR-138-5p/RGS5 axis and inhibited apoptosis, which could be a potential target for IH therapy.

## Figures and Tables

**Figure 1:** The flow chart of this study.

**Figure 2:** Analysis of hsa_circ_0003570, hsa-miR-138-5p, and *RGS5* mRNA expression levels in human dermal microvascular endothelial cells (HDMVECs) and hemangioma endothelial cells (HEMECs). (a) Binding sites' prediction of hsa_circ_0003570 and *RGS5* mRNA with hsa-miR-138-5p by the Encyclopedia of RNA Interactomes (ENCORI). (b) Quantitative real-time polymerase chain reaction (qRT-PCR) was used to detect the expression levels of hsa_circ_0003570, hsa-miR-138-5p, and *RGS5* mRNA in HDMVEC and HEMEC. ^∗^*p* < 0.05, compared with HDMVEC.

**Figure 3:** Silencing hsa_circ_0003570 inhibited the proliferation, migration, and invasion of HEMEC and promoted apoptosis. (a) The relative expression level of hsa_circ_0003570 to U6 was detected by quantitative real-time polymerase chain reaction (qRT-PCR) after no transfection group (control), no template control (si-NC), si-hsa_circ_0003570-1, si-hsa_circ_0003570-2, and si-hsa_circ_0003570-3 transfection. (b) The cell proliferation ability of HEMEC transfected with control, si-NC, and si-hsa_circ_0003570 was detected by MTT assay. (c) and (d) The cell migration ability and invasion ability of HEMEC transfected with control, si-NC, and si-hsa_circ_0003570 were detected by Transwell assay. (e) The apoptosis rate of HEMEC transfected with control, si-NC, and si-hsa_circ_0003570 was detected by flow cytometry. ^∗^*p* < 0.05, ^∗∗^*p* < 0.01, ^∗∗∗^*p* < 0.001, compared with control.

**Figure 4:** The effect of hsa_circ_0003570 on the malignant biological behavior of HEMEC cells could be reversed by hsa-miR-138-5p. (a) The expression levels of hsa_circ_0003570 and hsa-miR-138-5p in HEMEC transfected with no transfection group (control), no temple control (si-NC), si-hsa_circ_0003570, si-hsa_circ_0003570+hsa-miR-138-5p inhibitor, and hsa-miR-138-5p mimic were detected by quantitative real-time polymerase chain reaction (qRT-PCR). (b) The cell proliferation ability of HEMEC transfected with control, si-NC, si-hsa_circ_0003570, si-hsa_circ_0003570+hsa-miR-138-5p inhibitor, and hsa-miR-138-5p mimic was detected by MTT. (c) and (d) Cell migration and invasion ability of HEMEC transfected with control, si-NC, si-hsa_circ_0003570, si-hsa_circ_0003570+hsa-miR-138-5p inhibitor, and hsa-miR-138-5p mimic was detected by Transwell assay. (e) The apoptosis rate of HEMEC transfected with control, si-NC, si-hsa_circ_0003570, si-hsa_circ_0003570+hsa-miR-138-5p inhibitor, and hsa-miR-138-5p mimic was detected by flow cytometry. ^∗^*p* < 0.05, ^∗∗^*p* < 0.01, compared with Control.

**Figure 5:** hsa_circ_0003570, as the ceRNA of hsa-miR-138-5p, upregulated the expression of RGS5. (a) Putative miRNA binding sites in hsa_circ_0003570 and RGS5. (b) Putative miRNA binding sites in RGS5. (c) Detection of luciferase activity after hsa-miR-138-5p mimic and pGL3-hsa_circ_0003570 WT or pGL3-hsa_circ_0003570 MUT. (d) Luciferase activity detection after transfection with hsa-miR-138-5p mimic and pGL3-RGS5 WT or pGL3-RGS5 MUT. (e) Relative expression level of hsa_circ_0003570, hsa-miR-138-5p, and *RGS5* mRNA in HEMEC transfected with control, NC, si-hsa_circ_0003570, hsa-miR-138-5p mimic, si-hsa_circ_0003570+hsa-miR-138-5p inhibitor, and hsa-miR-138-5p inhibitor detected by qRT-PCR. (f) The relative expression of RGS5 in HEMEC after transfection with control, NC, si-hsa_circ_0003570, hsa-miR-138-5p mimic, si-hsa_circ_0003570+hsa-miR-138-5p inhibitor, and hsa-miR-138-5p inhibitor. ^∗^*p* < 0.05, compared with control.

**Figure 6:** RGS5 knockdown inhibited the proliferation, migration, and invasion of HEMEC cells and promoted apoptosis. (a) *RGS5* mRNA expression level of HEMEC transfected with after control, sh-NC, and sh-RGS5 was detected by qRT-PCR. (b) RGS5 protein expression level in HEMEC transfected with after control, sh-NC, and sh-RGS5 was detected by western blot. (c) The cell proliferation ability of HEMEC transfected with after control, sh-NC, and sh-RGS5 was detected by MTT assay. (d) and (e) The cell migration ability and invasion ability of HEMEC transfected with after control, sh-NC, and sh-RGS5 was detected by Transwell assay. (f) The apoptosis rate of HEMEC transfected with after control, sh-NC, and sh-RGS5 was detected by flow cytometry. ^∗^*p* < 0.05, ^∗∗^*p* < 0.01, ^∗∗∗^*p* < 0.001, ^∗∗∗∗^*p* < 0.0001, compare with control.

## Data Availability

The data used to support the findings of this study are available from the corresponding author upon request.

## Supplementary Materials

Supplementary Materials The following analysis results were based on the data from the GSE98795 dataset. Infantile hemangioma tumor tissue was obtained from 3 female patients 4-7 months old and 1 male patient 4 months old. The adjacent normal skin tissue was also obtained from 3 female patients 4-7 months old and 1 male patient 4 months old. The results of GEO2R analysis showed that a total of 234 circRNAs were upregulated and 374 circRNAs were downregulated (FC (abs) cut-off value 1.0) in the infantile hemangioma tumor tissue.
